The article "ITPKA expression is a novel prognostic factor in hepatocellular carcinoma" was published in 2015. Journal: Diagn Pathol.

# ITPKA expression is a novel prognostic factor in hepatocellular carcinoma

**DOI:** 10.1186/s13000-015-0374-1

**Published:** 2015-08-07

**Authors:** Jianbiao Li, Ying-Hui Zhu, Pinzhu Huang, Baozhu Zhang, Jian Sun, Xin-Yuan Guan

**Affiliations:** Sun Yat-sen University Cancer Center, State Key Laboratory of Oncology in South China, Collaborative Innovation Center for Cancer Medicine, Block 2, Room 708, 651 Dongfeng East Road, Guangzhou, 510060 China; Department of Clinical Oncology, The University of Hong Kong, L10-56, Laboratory Block, 21 Sassoon Road, Hong Kong, China; Department of Colorectal Surgery, The Sixth Affiliated Hospital, Sun Yat-sen University, Guangzhou, China

## Abstract

**Background:**

Inositol-1,4,5-trisphosphate-3-kinase-A (ITPKA) has recently been found to be implicated in the tumor progression of various cancers. However, the expression and the prognostic value of ITPKA in hepatocellular carcinoma (HCC) remains unexplored. The aim of this study is to investigate the clinical significance of ITPKA expression in HCC.

**Methods:**

We determined the expression level of ITPKA in 135 cases of HCC tissues and the matched adjacent nontumorous tissues by quantitative real-time RT-PCR. The correlation between ITPKA expression and prognosis of HCC patients was further evaluated by univariate and multivariate analysis. Multivariate analysis of the prognostic factors was performed with Cox proportional hazards model.

**Results:**

Up-regulation of ITPKA occurred in 48.9 % of primary HCCs compared with their nontumor counterparts (*P* < 0.001). In addition, high expression of ITPKA was significantly associated with vascular invasion (*P* = 0.001) and TNM stage (*P* = 0.005). Kaplan–Meier analysis showed that the 5-year overall survival (OS) and relapse-free survival (RFS) rate in the group with high expression of ITPKA is poorer than that in low expression group (32.2 and 26.8 % *versus* 59.2 and 57.7 %). Univariate and multivariate analyses revealed that ITPKA was an independent prognostic factor for OS and RFS. Moreover, Stratified analysis revealed that its prognostic significance still existed within the subgroup of patients with early clinical stage (TNM stage I) or normal serum AFP level (≤25 μg/L).

**Conclusion:**

Our data indicated that ITPKA expression was significantly up-regulated in HCC and could serve as a potential novel prognostic biomarker for HCC patients after surgery.

## Background

Hepatocellular carcinoma (HCC) is a highly lethal cancer, which has been ranked as the fifth most common malignancy and the third leading cause of cancer-related mortality worldwide [1–4]. Despite of the tremendous progress in diagnosis and multimodality treatment in the past decades, the prognosis of HCC patients remains grim, mainly because of its high recurrent and metastatic rate [5]. To date, numerous studies have identified a mass of dysregulated molecular events involved in liver carcinogenesis, which cover a wide range of genes with various functions. However, the biomarkers for HCC remain unsatisfactory in terms of high-risk population screening, clinical diagnosis and prognosis, and evaluation of treatment efficiency. Therefore, it is imperative to identify and characterize novel biomarkers for this disease.

The article "ITPKA expression is a novel prognostic factor in hepatocellular carcinoma" was published in 2015. Journal: Diagn Pathol.

With the advent of high-throughput sequencing technologies in recent years, transcriptome sequencing (RNA-Seq) has been a powerful tool for gene expression profiling in the study of cancer. Recently, our group exploited a RNA-Seq to delineate differential gene expression in ten pairs of HCC and nontumor clinical samples. Overexpression of inositol-1,4,5-trisphosphate-3-kinase-A (ITPKA) was observed in all ten HCC tumor tissues compared with their matched nontumoral counterparts. *ITPKA* gene, which is located in 15q15, encodes a predicted 461 amino acid polypeptide. Under physiological conditions, ITPKA is only identified in neurons and testis [6]. It is one of the three inositol trisphosphate 3-kinases (ITPKs) isoforms (A, B and C) that catalyse the phosphorylation of the second messenger inositol 1,4,5-trisphosphate (Ins(1, 4, 5)P_3_) to inositol 1, 3, 4, 5-tetrakisphosphate (Ins(1, 3, 4, 5)P_4_), and thus regulate Ins(1, 4, 5)P_3_-induced calcium (Ca^2+^) signals [7, 8]. Independent of this catalytic activity, ITPKA also binds and bundles filamentous actin (F-actin) to regulate the spine morphology [9]. Beside these physiological roles, ITPKA plays an important role in the carcinogenesis and metastasis. Down-regulated ITPKA expression was identified in oral squamous cell carcinoma (OSCC) tissues and OSCC cell lines [10]. Whereas in contrast, recent studies on lung cancer showed that high expression of ITPKA was detected in primary tumors and the matched lymph node metastases [11]. Furthermore, the analysis of RNA-seq data for kidney renal clear cell carcinoma patients showed that up-regulated ITPKA expression was associated with advanced stage and lower survival rates [12]. Taken together, we hypothesize that ITPKA may be a useful metastasis and prognostic marker for HCC.

In the present study, we investigated the expression levels of ITPKA in HCC and their paired adjacent nontumorous tissues, and further evaluated the correlation of ITPKA expression with clinical parameters and its prognostic value in HCC.

## Methods

### Patients and tissue samples

One hundred thirty five paired primary HCC tumor and nontumorous tissue samples were collected immediately after surgery resection at Sun Yat-sen University Cancer Center between December 2003 and September 2009. The enrollment criteria were as follows: (a) definitive HCC diagnosis by pathology based on WHO criteria; (b) no preoperative trans-hepatic arterial chemo-embolization or chemotherapy or radiotherapy before surgery; (c) surgical resection, defined as complete resection of all tumor nodules with the cut surface being free of cancer by histologic examination; (d) complete clinicopathologic and follow-up data. Ethical approval for this study was granted by the Medical Ethics Committee of Sun Yat-sen University Cancer Center. All patients signed informed consent. In this study, nontumoral liver tissues were defined as 2.0 cm from the tumor margin, which had been described previously [13]. Hepatitis B history was defined as history with positive serum hepatitis B surface antigen (HBsAg). Tumor encapsulation was defined as the presence of a clear fibrous sheath around the tumor at gross inspection. Tumor differentiation was based on the Edmondson and Steiner classification. HCC metastasis was defined as the presence of vascular invasion in the portal vein or the presence of satellite nodules surrounding a larger main tumor [14]. Tumor staging was determined according to the 7th edition tumor-node-metastasis (TNM) classification of the American Joint Committee on Cancer.

The article "ITPKA expression is a novel prognostic factor in hepatocellular carcinoma" was published in 2015. Journal: Diagn Pathol.

### Cell lines and culture conditions

HCC cell lines BEL7402, Hep3B, PLC8024, QSG7701, QGY7703, SMMC7721 and immortalized liver cell line LO2 were obtained from the Institute of Virology, Chinese Academy of Medical Sciences (Beijing, China). Huh7 was purchased from American type culture collection (ATCC, Manassas, Virginia, USA). Cells were maintained in high-glucose DMEM (Gibco BRL, Grand Island, NY) supplemented with 10 % fetal bovine serum (FBS) (Gibco BRL, Grand Island, NY). The cells were incubated at 37 °C in a humidified incubator containing 5 % CO_2_.

### Quantitative real-time reverse transcription polymerase chain reaction (qRT-PCR)

All fresh tumorous and nontumorous tissue samples were immediately stored at dry ice after resection and then frozen at −80 °C. Total RNA was extracted from clinical samples or cell lines using TRIzol reagent (Invitrogen), and was reverse-transcribed using an Advantage RT-for-PCR Kit (Clontech Laboratories) according to the manufacturer’s instructions. qRT-PCR was performed to detect levels of the corresponding glyceraldehyde-3-phosphate dehydrogenase (*GAPDH*) and *ITPKA* using a SYBR Green PCR Kit (Applied Biosystems) and LightCycler480 384-well PCR system (Roche Diagnostics). The *GAPDH* was used as an internal control for *ITPKA*. Primers for *ITPKA* are 5’-CCTTTCCACCTCGTCGGTCT-3’ (forward) and 5’-GCCTTAAAACTCCCAGTGTGC-3’ (reverse). Primers for *GAPDH* are 5’-ACTTCAACAGCGACACCCACTC-3’ (forward) and 5’-TACCAGGAAATGAGCTTGACAAAG-3’ (reverse). The value of relative expression for each sample was averaged and compared using the Ct method. ΔΔCt(sample) = ΔCt(sample) - ΔCt(calibrator), ΔCt(sample) = Ct(sample) of *ITPKA* - Ct(sample) of *GAPDH*; ΔCt(calibrator) = Ct(calibrator) of *ITPKA* - Ct(calibrator) of *GAPDH*; calibrator was defined as the pooled samples from 135 adjacent nontumorous tissues.

The article "ITPKA expression is a novel prognostic factor in hepatocellular carcinoma" was published in 2015. Journal: Diagn Pathol.

### Western blot analysis

ITPKA protein expression in cell lines was detected by Western blotting. Briefly, cells were washed twice with ice-cold PBS. Total protein was extracted with lysis buffer for 45 min on ice. Equal amounts of protein were separated by 12 % SDS-PAGE and electrophoretically transferred to polyvinylidene difluoride membranes (Millipore) using a mini trans-blot apparatus (Bio-Rad Laboratories). Membranes were blocked with PBS-0.05 % Tween 20 containing 5 % nonfat dry milk for one hour at room temperature and incubated with polyclonal rabbit anti-ITPKA (1:1,000; Proteintech) or monoclonal mouse anti-GAPDH antibody (1:5,000; Vazyme Biotech) at 4 °C overnight. Membranes were then washed three times with PBS-0.05 % Tween 20 and incubated with horseradish peroxidase–conjugated goat anti-rabbit or anti-mouse IgG (Santa Cruz Biotechnology) at a 1:5,000 dilution for one hour at room temperature. Blots were developed using an enhanced chemiluminescence kit (Pierce). Each experiment was repeated at least three times.

### Statistical analysis

All statistical analyses were performed using the Statistical Package for the Social Sciences (SPSS) version 16.0 (SPSS Inc, Chicago, IL). Paired two-tailed student’s *t* test was used to compare the expression of *ITPKA* in primary HCC tumors and their corresponding adjacent nontumorous tissues. The correlation between *ITPKA* expression and clinicopathological parameters was assessed by chi-square test or Fisher’s exact test. Disease-specific survival was calculated from the time of surgery to either the time of death from HCC or last follow up (31 December 2014). The prognostic value was calculated by the Kaplan-Meier analysis with log-rank test. Univariate and multivariate survival analysis was performed using the Cox proportional hazard model with a forward stepwise procedure (the entry and removal probabilities were 0.05 and 0.10, respectively). A significant difference was considered statistically when *P* value was <0.05.

## Results

### *ITPKA* expression was up-regulated in HCC

Our prior RNA-seq profiling data showed that *ITPKA* was overexpressed in all ten tested HCC tumor tissues. High expression of *ITPKA* (defined as > 2-fold change) was detected in 66 of 135 (48.9 %) of HCC tissues by qRT-PCR, compared with their normal counterparts. The average level of *ITPKA* expression in tumor tissues was significantly higher than that in non-tumor tissues (1.11 *versus* 3.01, *P* < 0.001, paired Student’s *t* test; Fig. 1a). The median fold change of *ITPKA* (1.84) in HCC tumor tissues was used as a cutoff value to divide all 135 patients into two groups: the high expression group (*n* = 66) and the low expression group (*n* = 69). The expression levels of ITPKA in seven HCC cell lines and one immortalized liver cell line (LO2) were tested by qRT-PCR and western blot analysis. Compared with LO2, up-regulation of ITPKA was detected in QGY7703, Hep3B, Huh7 and PLC8024 cells (Fig. 1b).

The article "ITPKA expression is a novel prognostic factor in hepatocellular carcinoma" was published in 2015. Journal: Diagn Pathol.

**Fig. 1:** *ITPKA* was up-regulated in HCCs. **a** *ITPKA* mRNA was markedly increased in tumor tissues than that in the paired adjacent nontumor tissues. **, *P* < 0.001, paired *t*-test. **b** Up-regulation of ITPKA was detected in 4 of 7 HCC cell lines by qRT-PCR (*upper*) and western blot analysis (*lower*). Immortalized liver cell line (LO2) was used as control

### Clinicopathologic features of *ITPKA* in HCC patients

The correlation between *ITPKA* mRNA expression in primary HCC and clinicopathological features was summarized in Table 1. High expression of *ITPKA* was significantly associated with vascular invasion (*P* = 0.001) and TNM stage (*P* = 0.005). No correlation was observed between *ITPKA* expression and other clinicopathological characteristics.

**Table 1:** Association of *ITPKA* expression with clinicopathological features in HCCs

Clinical features	Cases	*ITPKA* expression		*P* value
		low level (%)	high level (%)	
Age (years old)				0.945
≤50	63	32 (50.8 %)	31 (49.2 %)	
>50	72	37 (51.4 %)	35 (48.6 %)	
Gender				1.000
Male	128	65 (50.8 %)	63 (49.2 %)	
Female	7	4 (57.1 %)	3 (42.9 %)	
HBsAg				0.201
Negative	15	10 (66.7 %)	5 (33.3 %)	
Positive	120	59 (49.2 %)	61 (50.8 %)	
AFP (μg/L)				0.212
≤25	48	28 (58.3 %)	20 (41.7 %)	
>25	87	41 (47.1 %)	46 (52.9 %)	
Cirrhosis				0.569
No	23	13 (56.5 %)	10 (43.5 %)	
Yes	112	56 (50.0 %)	56 (50.0 %)	
Tumor size (cm)				0.126
≤5	56	33 (58.9 %)	23 (41.1 %)	
>5	79	36 (45.6 %)	43 (54.4 %)	
Tumor number				0.116
Solitary	104	57 (54.8 %)	47 (45.2 %)	
Multiple	31	12 (38.7 %)	19 (61.3 %)	
Tumor encapsulation				0.455
Complete	43	24 (55.8 %)	19 (44.2 %)	
None	92	45 (48.9 %)	47 (51.1 %)	
Vascular invasion				**0.001**
Absent	114	65 (57.0 %)	49 (43.0 %)	
Present	21	4 (19.0 %)	17 (81.0 %)	
Edmondson-Steiner				0.106
I-II	79	45 (57.0 %)	34 (43.0 %)	
III-IV	56	24 (42.9 %)	32 (57.1 %)	
TNM stage				**0.005**
I	93	55 (59.1 %)	38 (40.9 %)	
II-III	42	14 (33.3 %)	28 (66.7 %)	

Statistical significance (*P* < 0.05) is shown in bold

The article "ITPKA expression is a novel prognostic factor in hepatocellular carcinoma" was published in 2015. Journal: Diagn Pathol.

### Association between *ITPKA* expression and patient survival

Univariate analysis showed that HBsAg, serum AFP level, tumor size, tumor number, vascular invasion, TNM stage, and *ITPKA* expression were prognostic factors for OS and RFS (Table 2). The 5-year OS and RFS rate in the high *ITPKA* expression group were significantly lower than those in the low *ITPKA* expression group (32.2 and 26.8 % *versus* 59.2 and 57.7 %; Fig. 2a). Considering that the TNM stage was correlated with several clinical indexes (such as tumor size, tumor number, and vascular invasion), we did not introduce it into the multivariate Cox proportional hazard model to avoid potential bias. The multvariate analysis demonstrated that *ITPKA* expression, HBsAg and vascular invasion were independent prognostic predictors for RFS (Table 3). Further, in a stratified survival analysis according to the TNM stage or serum AFP level, we found that the prognostic significance of *ITPKA* was retained in TNM stage I (*P* = 0.001), normal AFP level (≤25 μg/L; *P* = 0.047) and high AFP level (>25 μg/L; *P* = 0.001) subgroups (Fig. 2b and c).

**Table 2:** Univariate Cox regression analyses for OS and RFS in HCCs

Clinical features	OS		RFS	
	HR (95 % CI)	*P* value	HR (95 % CI)	*P* value
Age	0.678 (0.420–1.096)	0.113	0.653 (0.409–1.041)	0.073
Gender	2.297 (0.562–9.390)	0.247	2.526 (0.619–10.316)	0.197
HBsAg	3.379 (1.061–10.763)	**0.039**	3.581 (1.126–11.394)	**0.031**
AFP	2.187 (1.246–3.839)	**0.006**	2.000 (1.171–3.418)	**0.011**
Cirrhosis	1.025 (0.549–1.916)	0.937	1.127 (0.605–2.097)	0.707
Tumor size	2.161 (1.279–3.653)	**0.004**	1.870 (1.135–3.081)	**0.014**
Tumor number	2.475 (1.488–4.118)	<**0.001**	2.576 (1.574–4.216)	<**0.001**
Tumor encapsulation	0.674 (0.392–1.161)	0.155	0.722 (0.429–1.215)	0.221
Vascular invasion	6.074 (3.449–10.698)	<**0.001**	5.722 (3.236–10.119)	**<0.001**
Edmondson-Steiner	1.348 (0.832–2.186)	0.225	1.296 (0.810–2.074)	0.279
TNM stage	4.919 (3.014–8.082)	<**0.001**	4.282 (2.654–6.907)	**<0.001**
*ITPKA* expression	2.579 (1.567–4.245)	<**0.001**	2.669 (1.638–4.349)	**<0.001**

*HR* hazard ratio; *CI* confidence interval; statistical significance (*P* < 0.05) is shown in bold

**Fig. 2:** Kaplan-Meier analysis of OS and RFS for *ITPKA* expression. **a** Kaplan-Meier analysis of OS and RFS for *ITPKA* expression in 135 cases of HCC patients. **b** Stratified survival analysis according to the TNM stage. **c** Stratified survival analysis according to the serum AFP level

**Table 3:** Multivariate Cox regression analyses for OS and RFS in HCCs

Clinical features	OS		RFS	
	HR (95 % CI)	*P* value	HR (95 % CI)	*P* value
HBsAg	3.262 (0.999–10.645)	0.050	3.330 (1.022–10.849)	**0.046**
AFP	1.477 (0.810–2.695)	0.203	1.376 (0.777–2.436)	0.273
Tumor size	1.939 (1.106–3.399)	**0.021**	1.624 (0.949–2.780)	0.077
Tumor number	1.348 (0.763–2.383)	0.304	1.469 (0.841–2.566)	0.176
Vascular invasion	3.325(1.752–6.309)	<**0.001**	2.917 (1.533–5.553)	**0.001**
*ITPKA* expression	1.825 (1.064–3.132)	**0.029**	1.868 (1.099–3.175)	**0.021**

*HR* hazard ratio; *CI* confidence interval; statistical significance (*P* < 0.05) is shown in bold

The article "ITPKA expression is a novel prognostic factor in hepatocellular carcinoma" was published in 2015. Journal: Diagn Pathol.

## Discussion and conclusions

The intracellular second messenger Ins(1,4,5)P_3_ controls many different cellular functions by regulating internal Ca^2+^ signals [7]. The lifetime of Ins(1,4,5)P_3_ is tightly regulated by two mechanisms: phosphorylation *via* ITPKs to Ins(1,3,4,5)P_4_ or dephosphorylation *via* ins(1,4,5)P_3_ 5-phosphatase (INPP5A) to inositol 1,4-bisphosphate (Ins(1,4)P_2_) [15, 16]. ITPKA is the most highly characterized ITPKs isoform, and found up-regulated in lung cancer tumor tissues [11]. In the present study, our data demonstrated that 48.9 % of HCC patients showed elevated *ITPKA* expression in their tumorous specimens compared with their normal counterparts. However, down-regulation of ITPKA was found in oral squamous cell carcinoma, suggesting that ITPKA may serve as a tumor-suppressor [10]. Based on these studies, the function of ITPKA seems to depend on its cellular context.

We next investigated the clinicopathologic correlation of *ITPKA* expression in HCC patients. The results showed that overexpression of *ITPKA* correlated with vascular invasion (*P* = 0.001) and TNM stage (*P* = 0.005), which strongly suggested that ITPKA was involved in the metastasis and progression of HCC. This is in an agreement with two recent studies, which showed that ectopic expression of ITPKA enhanced the metastatic potential of tumor cells [11, 17]. Ca^2+^ is a ubiquitous second messenger that mediates numerous cellular processes, including cell proliferation, survival, apoptosis, migration and gene expression. Increases of intracellular Ca^2+^ concentration have long been known to be involved in cell migration and invasion. Ins(1,4,5)P_3_ can bind to the ER membrane Ca^2+^-permeable Ins(1,4,5)P_3_ receptor (IP_3_R) channels, which results in the opening of the membrane channel, and further release the stored Ca^2+^ into the cytosol [18, 19]. ITPKA metabolizes Ins(1,4,5)P_3_ to Ins(1,3,4,5)P_4_, which in turn terminates the signal to release Ca^2+^ from the endoplasmic reticulum. On the other hand, in some cases the Ins(1,3,4,5)P_4_, generated by ITPKA, can protect Ins(1,4,5)P_3_ by competitively inhibiting the activity of INPP5A and thus prolongs the effect of Ins(1,4,5)P_3_ on Ca^2+^ signals [20, 21]. Moreover, a recent report demonstrated that in EGF-stimulated tumor cells Ins(1,3,4,5)P_4_ prolonged Ca^2+^ signaling by activation of SOCE [17]. Hence, we speculated that ITPKA might enhance the metastatic potential of HCC cells by increasing intracellular Ca^2+^ concentration. However, further studies are required to elucidate the function and mechanisms of ITPKA that involved in the Ca^2+^ signaling in HCC. During metastatic dissemination, cancer cells must acquire the ability to migrate, which is correlated with cytoskeletal remodeling. Independent of its InsP_3_ kinase activity, ITPKA can modify spine shape and internal microstructure by directly binding and bundling actin filaments and/or by recruiting Rac1 and associated signaling machinery [9, 22]. It has also been shown that ITPKA induces the formation of filopodia- and lamellipodia-like protrusions, and consequently enhances the migratory and invasive abilities of tumor cells [17, 23]. Consequently, the migration-promoting effect of ITPKA is regulated by both enzyme activity-dependent and activity-independent mechanism. Besides, Ins(1,3,4,5)P_4_ itself has the potential to regulate various cellular functions by acting on multiple targets, the majority of which contain pleckstrin homology (PH) domains [24]. One of earliest suggested Ins(1,3,4,5)P_4_ effectors are channel proteins residing in the plasma membrane. For example, Ins(1,3,4,5)P_4_ can activate K^+^ channels in the plasma membrane in cooperation with the internal Ca^2+^ [25]. In mouse lacrimal acinar cell, Ca^2+^-dependent Cl-channel is also implicated as a Ins(1,3,4,5)P_4_ effector [26]. The second major class of Ins(1,3,4,5)P_4_ effectors are regulators of the small G proteins Ras and Rap. Ins(1,3,4,5)P_4_ plays contradicting roles in different models: Ins (1,3,4,5) P_4_ promotes the activation of a unique Ras-GAP (GAP1^IP4BP^), and consequently inactivation of the Ras GTPase; or inhibits RASA3 GAP activity by removing RASA3 from the plasma membrane [27–29]. Nevertheless, until now, the components of Ins(1,3,4,5)P_4_-based signaling systems are far from clear. Further studies are required to define the roles of ITPKA and its products precisely in HCC.

The article "ITPKA expression is a novel prognostic factor in hepatocellular carcinoma" was published in 2015. Journal: Diagn Pathol.

Our study also demonstrated that high expression of *ITPKA* was one of the most important prognosis factors for OS and RFS in the univariate and multivariate analysis. The 5-year RFS of patients with high *ITPKA* expression was markedly shorter than that with low expression (26.8 % *versus* 57.7 %). It is known that HCC patients with the same TNM stage, histopathologic features of tumor, and treatment strategy (such as curative resection) may experience quite different clinical outcomes [30]. With the stratified survival analysis according to the TNM stage, we found that the prognostic significance of *ITPKA* still existed in subgroup of patients in early clinical stage (TNM stage I): the 5-year RFS for *ITPKA* high expression and low expression patients was 40.0 % *versus* 72.1 % (*P* = 0.001). AFP is the current gold standard and most commonly used biomarker for the diagnosis and monitoring the effectiveness of treatment or recurrence in HCC patients [31]. Until now, there was no ideal biomarker for monitoring recurrence and metastasis in HCC patients with normal AFP level after curative resection [32, 33]. Interestingly, we found that *ITPKA* status could stratified the normal AFP level group into two subgroups with substantially different 5-year RFS (29.3 and 74.2 % for *ITPKA* high and low patients, respectively; *P* = 0.047). Given that there were only 48 cases of HCC patients with normal AFP level in the present study, further investigation with a larger sample size is required to confirm this finding.

In conclusion, the results of present study for the first time demonstrated that high expression of *ITPKA* in HCC tumorous specimens indicated aggressive tumor behaviors and predicted a poor clinical outcome. These findings suggested that *ITPKA* may serve as a suitable prognostic marker for HCC patients after surgery, especially in early clinical stage.

## Abbreviations

ITPKA: Inositol-1,4,5-trisphosphate-3-kinase-A
HCC: Hepatocellular carcinoma
OS: Overall survival
RFS: Relapse-free survival
AFP: Alpha-fetoprotein
TNM: Tumor Node Metastasis
RNA-Seq: Transcriptome sequencing
ITPKs: Trisphosphate 3-kinases
Ins(1,4,5)P_3_: Inositol 1,4,5-trisphosphate
Ins(1,3,4,5)P_4_: Inositol 1,3,4,5-tetrakisphosphate
INPP5A: Ins(1,4,5)P_3_ 5-phosphatase
Ins(1,4)P_2_: Inositol 1,4-bisphosphate
Ca^2+^: Calcium
F-actin: Filamentous actin
OSCC: Oral squamous cell carcinoma
qRT-PCR: Quantitative real-time reverse transcription polymerase chain reaction
PH: Pleckstrin homology
GAPDH: Glyceraldehyde-3-phosphate dehydrogenase
